RETRACTED

# Doripenem, Ertapenem, and Meropenem Sensitivity in Salmonella Typhi: A Cross-Sectional Study From Pakistan

**DOI:** 10.7759/cureus.72872

**Published:** 2024-11-02

**Authors:** Mian Mufarih Shah, Imran Khan, Mehwash Iftikhar, Nazir Shah, Saeed Ur Rahman, Jahanzeb Khan

**Affiliations:** 1 Department of Medicine, Medical Teaching Institution (MTI) Hayatabad Medical Complex, Peshawar, PAK; 2 Department of Internal Medicine, Hayatabad Medical Complex, Peshawar, PAK; 3 Department of Medicine, Hayatabad Medical Complex, Peshawar, PAK; 4 Department of Pathology, Khyber Girls Medical College, Peshawar, PAK; 5 Department of Microbiology, Hayatabad Medical Complex, Peshawar, PAK; 6 Department of Pharmacy, Hayatabad Medical Complex, Peshawar, PAK

**Keywords:** doripenem, ertapenem, meropenem, multidrug-resistant pathogen, salmonella typhi

## Abstract

Background

*Salmonella *Typhi (*S. *Typhi) is increasingly resistant to multiple antibiotics, posing a challenge in treatment, particularly in multidrug-resistant (MDR) cases. Carbapenems, including doripenem, ertapenem, and meropenem, have been considered last-resort options. This study evaluates the effectiveness of these carbapenems against *S. *Typhi isolates in a clinical setting in Peshawar, Pakistan.

Objective

To assess the effectiveness of the carbapenem antibiotics, doripenem, ertapenem, and meropenem, against *S. *Typhi.

Methods

This study collected data from blood cultures of patients diagnosed with *S. *Typhi infections at the Hayatabad Medical Complex in Peshawar, Pakistan for two years: from January 1, 2022, to December 31, 2023. Sensitivity testing was performed using the disk diffusion method in accordance with Clinical and Laboratory Standards Institute (CLSI) guidelines. The analysis examined the sensitivity rates of the three antibiotics and compared their effectiveness.

Results

A total of 626 *S. *Typhi isolates were tested. Only 11.98% of the isolates were sensitive to doripenem, while 88.02% were resistant to it. In contrast, 35.5% of the isolates responded to ertapenem, with 64.5% being resistant. Meropenem showed the highest efficacy, with 42.7% of the isolates demonstrating sensitivity. These findings highlight the growing challenge of managing multidrug-resistant (MDR) *S. *Typhi infections, especially in regions where resistance to carbapenems is becoming prevalent.

Conclusion

Meropenem proved to be more effective against *S. *Typhi compared to doripenem and ertapenem. The study emphasizes the need for ongoing monitoring of resistance patterns and the exploration of alternative or combination treatment options. These findings have immediate clinical implications for empiric therapy choices and highlight the urgent need for antibiotic stewardship programs in endemic regions.

RETRACTED

## Introduction

*Salmonella *Typhi (*S. *Typhi), is a Gram-negative, obligatory anaerobic bacterium. It belongs to the serogroup D within subspecies I of the genus *Salmonella*. It is responsible for typhoid fever, which causes around 11-21 million cases and 128,000-161,000 deaths globally each year [1].

The selection of the three carbapenems, doripenem, ertapenem, and meropenem, for this study, was based on their distinct clinical applications and characteristics. Meropenem has established itself as the preferred choice for severe infections due to its broad spectrum and documented safety profile. Ertapenem provides the advantage of once-daily dosing, making it particularly suitable for outpatient settings. Doripenem has shown promising results against resistant Gram-negative organisms in recent clinical investigations. Understanding the comparative effectiveness of these antibiotics is crucial for optimizing treatment protocols in clinical settings. The resistance patterns observed are particularly concerning, as similar trends have been documented even in non-clinical settings, including poultry populations [2,3].

Typhoid fever disproportionately affects low- and middle-income countries as classified by World Bank criteria, particularly in regions with limited healthcare infrastructure and inadequate water and sanitation facilities. The emergence and spread of multidrug-resistant (MDR) strains of *S. *Typhi have significantly complicated treatment protocols, leading to increased morbidity and mortality rates [1]. Recent surveillance data from Pakistan has revealed an alarming increase in the prevalence of MDR *S. *Typhi strains, creating significant therapeutic challenges [4].

The situation in resource-limited countries is particularly concerning, as treatment options become increasingly limited. Healthcare providers face mounting challenges as the number of MDR cases continues to rise, necessitating the exploration of various antibiotic combinations. The therapeutic options are not exhaustive, and these regions face an unprecedented threat of extensive drug resistance (XDR) [4].

The global proliferation of MDR *S. *Typhi represents a critical public health challenge. Traditional treatment approaches have become increasingly ineffective, with fluoroquinolones, once considered reliable first-line treatments, now showing limited efficacy even in uncomplicated cases. The situation is particularly dire in regions with high rates of antibiotic misuse, where oral medications have become largely ineffective [4]. Research by Ali Shah et al. has demonstrated that over 70% of *S.* Typhi isolates in Pakistan now show resistance to fluoroquinolones, emphasizing the urgent need for alternative treatment strategies [5].

RETRACTED

The effectiveness of third-generation cephalosporins, particularly ceftriaxone, has also diminished significantly due to the emergence of extended-spectrum beta-lactamase (ESBL)-producing strains of *S. *Typhi [6]. In this context, carbapenems, including doripenem, meropenem, and ertapenem, have emerged as critical last-resort options for treating MDR Gram-negative bacterial infections [7]. These medications are typically reserved for severe cases where other treatment options have proven ineffective [8].

Recent research by Qureshi et al. has demonstrated meropenem's superior efficacy against resistant Gram-negative bacteria, including *S. *Typhi [9]. However, the emergence of carbapenem resistance, particularly in South Asia, presents a new challenge to effective treatment [10]. Studies by Yousaf et al. have documented decreasing effectiveness of doripenem in Pakistan, with resistance rates reaching as high as 88% [11]. The resistance patterns extend beyond carbapenems, with high resistance rates also observed for cephalosporins and azithromycin [12]. Among the carbapenems, meropenem continues to demonstrate superior effectiveness in treating *S. *Typhi, particularly in cases involving severe infections and high-level resistance [13].

The present study was designed to evaluate the comparative effectiveness of these three carbapenem antibiotics against *S. *Typhi isolates in a clinical setting in Peshawar, Pakistan. This research aims to provide evidence-based guidance for clinicians treating MDR *S. *Typhi infections and contribute to the ongoing surveillance of antimicrobial resistance patterns in the region.

## Materials and methods

Study design and setting

This cross-sectional study was conducted using clinical data from blood cultures of patients diagnosed with *S.* Typhi at Hayatabad Medical Complex in Peshawar, Pakistan, using a consecutive sampling technique. The study received ethical approval (approval no. 2222, dated December 8, 2021) from the ethical approval committee of Hayatabad Medical Complex, Peshawar, before study initiation. The investigation spanned two years, from January 1, 2022, to December 31, 2023.

Patient selection and sample collection

The study population comprised culture-positive patients diagnosed with typhoid fever who were above 12 years of age, encompassing both male and female patients. The exclusion criteria were carefully defined to ensure data quality: patients showing clear evidence of other infections were excluded, as were those whose blood cultures revealed *Salmonella* Paratyphi strains. Blood sample collection followed strict sterile procedures, with 8-10 ml of venous blood drawn and inoculated into specialized blood culture bottles (Bactec™ Plus Aerobic, Anaerobic, Becton Dickinson, Franklin Lakes, NJ, USA) containing 30 ml of broth.

RETRACTED

Laboratory procedures

Sample processing was conducted using the Bactec™ FX-40 system (Becton Dickinson, Franklin Lakes, NJ, USA). Upon detection of positive cultures, subsequent subculturing was performed on McConkey and blood agar (Oxoid™, Basingstoke, UK), with incubation maintained at 35 ± 2°c for 24 hours following standard protocols. Serotype identification was accomplished using group- and type-specific antisera (Bio-Rad, Hercules, CA, USA).

Antibiotic sensitivity testing

Antibiotic sensitivity assessment was performed using the disk diffusion method, adhering strictly to Clinical and Laboratory Standards Institute (CLSI) M100-ED33:2023 guidelines [14]. The testing protocol utilized standard antibiotic disks from Oxoid™ (Basingstoke, UK) or Hardy Diagnostics (Santa Maria, CA, USA), with each antibiotic (doripenem, ertapenem, and meropenem) administered at a concentration of 10 µg. Environmental conditions for disk storage were maintained at 2-8°C, with manufacturer-provided desiccant to ensure stability. Quality assurance was maintained through regular testing with *Escherichia coli* ATCC® 25922™ (ATCC, Manassas, VA, USA) reference strain.

Sensitivity interpretation followed CLSI M100-ED33:2023 breakpoint criteria. For carbapenems, isolates were classified as sensitive or resistant based on the following zone diameter breakpoints: doripenem (sensitive ≥23 mm, resistant ≤19 mm), ertapenem (sensitive ≥22 mm, resistant ≤18 mm), and meropenem (sensitive ≥23 mm, resistant ≤19 mm). Intermediate readings were classified as resistant for analysis purposes.

Quality assurance protocols

A comprehensive quality control system was implemented throughout the study period. This system encompassed regular visual inspections of mueller-hinton agar plates, systematic sterility verification of media, and strict maintenance of standardized incubation conditions at 35°C ± 2°C. Temperature monitoring and incubator maintenance were performed regularly. Zone measurements were conducted by trained laboratory technologists under direct supervision of senior microbiologists. The laboratory maintained quality standards through both internal quality checks and participation in external quality assurance programs when available.

Data collection and management

A comprehensive data collection protocol was implemented using a standardized form designed specifically for this study. Patient demographics were systematically documented, encompassing age, gender, and residential categorization between urban and rural areas. The clinical profile documentation included detailed medical history, with particular attention to previous antibiotic usage patterns and existing comorbidities. Disease progression indicators were carefully recorded, including the severity of presenting symptoms, their duration, and the total length of hospital stay. The laboratory component of data collection focused on culture results, with detailed documentation of antibiotic sensitivity patterns and precise measurements of inhibition zones. All collected data were entered into a secure, password-protected database with regular automated backup systems in place to ensure data integrity and confidentiality.

RETRACTED

Statistical analysis

Data analysis was performed using IBM SPSS Statistics for Windows, version 26 (IBM Inc., Armonk, NY, USA). The analytical approach began with descriptive statistics for demographic and clinical characteristics. For categorical variables, frequencies and percentages were computed, while means and standard deviations were calculated for continuous variables. The comparative analysis of antibiotic sensitivity rates employed Chi-square tests, with statistical significance determined at p < 0.05. The relationship between demographic factors and antibiotic resistance was assessed through odds ratios (OR) with corresponding 95% confidence intervals (CI).

Ethical considerations

The study protocol adhered comprehensively to the ethical principles outlined in the Declaration of Helsinki. Written informed consent was obtained from all study participants or their legal guardians prior to enrollment. Patient confidentiality was maintained throughout the study through the use of coded identifiers in all documentation. The complete study protocol underwent review and received approval from the institutional ethics committee, with all procedures conducted in accordance with the institution's established guidelines for research involving human subjects.

## Results

This study evaluated the sensitivity of *S.* Typhi isolates to three carbapenem antibiotics: doripenem, ertapenem, and meropenem. A total of 626 isolates were tested to determine their response rates. The analysis encompassed both the demographic characteristics of the study population and their association with carbapenem resistance patterns.

The demographic and clinical characteristics of the study population demonstrated several significant associations with carbapenem resistance, as presented in Table 1. Age distribution analysis revealed that the majority of patients fell within the 20-30-year age range, comprising 61.5% of the total study population. The age-specific resistance patterns showed higher resistance rates among younger patients, with those aged 21-30 years demonstrating the highest resistance rate of 85.4% (OR: 2.67, 95% CI: 1.68-4.25, p<0.001).

RETRACTED

**Table 1:** Demographic and clinical characteristics associated with carbapenem resistance. χ²: Chi-square, p-value: statistical significance.

Characteristic	Total N (%)	Resistant N (%)	Sensitive N (%)	OR (95% CI)	χ² value	p-value
Age (years)						
0-20	187 (29.9)	156 (83.4)	31 (16.6)	2.31 (1.45-3.68)	12.43	0.001
21-30	198 (31.6)	169 (85.4)	29 (14.6)	2.67 (1.68-4.25)	16.82	<0.001
31-40	142 (22.7)	108 (76.1)	34 (23.9)	1.46 (0.89-2.39)	2.25	0.134
41-50	67 (10.7)	46 (68.7)	21 (31.3)	1.00 (Ref)	-	-
>50	32 (5.1)	20 (62.5)	12 (37.5)	0.76 (0.32-1.81)	0.38	0.537
Gender						
Male	358 (57.2)	285 (79.6)	73 (20.4)	1.05 (0.73-1.52)	-	-
Female	268 (42.8)	211 (78.7)	57 (21.3)	1.00 (Ref)	-	-
Location						
Urban	389 (62.1)	331 (85.1)	58 (14.9)	2.34 (1.62-3.38)	-	-
Rural	237 (37.9)	165 (69.6)	72 (30.4)	1.00 (Ref)	-	-
Prior antibiotics						
None	142 (22.7)	82 (57.7)	60 (42.3)	1.00 (Ref)	-	-
Single	247 (39.5)	197 (79.8)	50 (20.2)	2.89 (1.84-4.54)	21.47	<0.001
Multiple	237 (37.8)	217 (91.6)	20 (8.4)	7.93 (4.52-13.91)	58.31	<0.001
Comorbidities						
None	412 (65.8)	308 (74.8)	104 (25.2)	1.00 (Ref)	-	-
Diabetes	87 (13.9)	79 (90.8)	8 (9.2)	3.33 (1.58-7.02)	9.87	0.002
Hypertension	56 (8.9)	45 (80.4)	11 (19.6)	1.38 (0.68-2.81)	0.79	0.374
Other	71 (11.4)	64 (90.1)	7 (9.9)	3.08 (1.38-6.87)	7.62	0.006
Severity						
Mild	198 (31.6)	138 (69.7)	60 (30.3)	1.00 (Ref)	-	-
Moderate	289 (46.2)	234 (81.0)	55 (19.0)	1.85 (1.23-2.79)	8.89	0.003
Severe	139 (22.2)	124 (89.2)	15 (10.8)	3.59 (1.95-6.61)	17.43	<0.001
Illness duration						
<1 week	187 (29.9)	127 (67.9)	60 (32.1)	1.00 (Ref)	-	-
1-2 weeks	328 (52.4)	271 (82.6)	57 (17.4)	2.25 (1.49-3.39)	15.26	<0.001
>2 weeks	111 (17.7)	98 (88.3)	13 (11.7)	3.57 (1.89-6.75)	15.89	<0.001
Hospital stay						
Outpatient	198 (31.6)	138 (69.7)	60 (30.3)	1.00 (Ref)	-	-
<7 days	267 (42.7)	216 (80.9)	51 (19.1)	1.84 (1.22-2.78)	8.52	0.004
7-14 days	124 (19.8)	108 (87.1)	16 (12.9)	2.93 (1.64-5.24)	13.24	<0.001
>14 days	37 (5.9)	34 (91.9)	3 (8.1)	4.93 (1.47-16.54)	6.64	0.010

Detailed analysis of demographic factors revealed significant patterns in antibiotic sensitivity. Age-stratified analysis showed higher resistance rates in younger patients (21-30 years), possibly reflecting greater healthcare exposure or antibiotic use in this age group. While gender didn't significantly influence resistance patterns (p=0.782), infection severity correlated strongly with resistance profiles. Severe infections showed higher resistance rates (89.2%) compared to moderate (81.0%) and mild cases (69.7%), suggesting a potential relationship between disease severity and antibiotic resistance development. Urban residents demonstrated significantly higher resistance rates (85.1%) compared to rural residents (69.6%), highlighting the potential impact of healthcare access and antibiotic use patterns on resistance development (Table 1).

RETRACTED

Gender distribution analysis showed a slight male predominance (57.2%) in the study population. However, gender did not demonstrate a statistically significant association with carbapenem resistance (p=0.782). Urban residents showed significantly higher resistance rates (85.1%) compared to rural residents (69.6%), with an OR of 2.34 (95% CI: 1.62-3.38, p<0.001).

Prior antibiotic exposure significantly influenced resistance patterns. Patients with multiple previous antibiotic exposures showed the highest resistance rates (91.6%), compared to those with single antibiotic exposure (79.8%) and no prior antibiotic use (57.7%). This trend demonstrated a clear dose-response relationship (p<0.001).

The severity of illness also correlated with resistance patterns. Severe cases showed higher resistance rates (89.2%) compared to moderate (81.0%) and mild cases (69.7%). Similarly, longer illness duration was associated with increased resistance, with patients ill for more than two weeks showing the highest resistance rates (88.3%).

Hospital stay duration analysis revealed a progressive increase in resistance rates with longer stays. Outpatients showed the lowest resistance rates (69.7%), while those hospitalized for more than 14 days demonstrated the highest resistance (91.9%), suggesting a potential relationship between healthcare exposure and resistance development.

The analysis of antibiotic sensitivity patterns revealed varying degrees of effectiveness among the three tested carbapenems (Table 2).

**Table 2:** Sensitivity of S. Typhi to doripenem, ertapenem, and meropenem. OR: odds ratio, CI: confidence interval, χ²: Chi-square value, p-value: statistical significance.

Antibiotic	Sensitive N (%)	Resistant N (%)	p-value (compared to meropenem)
Doripenem	75 (11.98)	551 (88.02)	<0.05
Ertapenem	222 (35.50)	404 (64.50)	>0.05
Meropenem	267 (42.70)	359 (57.30)	-

Meropenem demonstrated the highest efficacy with a sensitivity rate of 42.70%. This was followed by ertapenem, which showed moderate effectiveness with 35.50% sensitivity. Doripenem exhibited the lowest sensitivity at 11.98%, with a corresponding high resistance rate of 88.02%. The difference in effectiveness between doripenem and meropenem was statistically significant (p < 0.05), while the difference between ertapenem and meropenem did not reach statistical significance (p > 0.05).

RETRACTED

## Discussion

The present study provides important insights into the effectiveness of three commonly used carbapenem antibiotics against *S.* Typhi in a clinical setting. The findings reveal that meropenem demonstrated the highest efficacy (42.7% sensitivity) among the tested carbapenems, followed by ertapenem (35.5%) and doripenem (11.98%). These results align with previous research by Yousaf et al., who documented meropenem's superior effectiveness in adolescents, and Ullah et al. who documented this in children [11,15]. Furthermore, research conducted in Pakistan by Jabeen et al. has confirmed meropenem's position as the preferred treatment for MDR *Salmonella*, citing its broad-spectrum activity and consistent effectiveness against resistant strains [16].

The clinical implications of these resistance patterns are significant. The high resistance rate to doripenem (88.02%) suggests its use may lead to treatment failures and potentially worse clinical outcomes. This finding necessitates a reconsideration of current treatment guidelines, particularly in regions where doripenem is commonly prescribed. The moderate effectiveness of ertapenem (35.5% sensitivity) indicates its role might be limited to carefully selected cases with confirmed sensitivity. Our findings support the implementation of robust antibiotic stewardship programs, which should include regular monitoring of resistance patterns, restriction of carbapenem use to confirmed sensitive cases, implementation of pre-authorization requirements for carbapenem prescriptions, and regular physician education about resistance patterns. These measures could help preserve the effectiveness of remaining sensitive antibiotics.

The poor performance of doripenem, evidenced by its 88.02% resistance rate, raises significant concerns about its continued utility in treating *S.* Typhi infections. This finding corresponds with observations by Bhutta et al., who documented a marked decline in doripenem's efficacy across South Asia [17]. The implications of this high resistance rate suggest that doripenem may no longer be a viable treatment option in regions where MDR *Salmonella *strains are prevalent [18]. While ertapenem showed better results than doripenem, its effectiveness as monotherapy for MDR infections remains limited due to its narrower spectrum of activity, as previously documented by Mahmood et al. [10].

The observed resistance patterns extend beyond South Asia, though with varying intensity. Research from Africa and the Middle East has reported increasing resistance rates, albeit lower than those observed in South Asian populations [7]. The findings from Pakistan by Mahmood et al. parallel our results, showing the maintained effectiveness of meropenem while documenting increasing resistance to doripenem, consistent with patterns reported by Jabeen et al. and Mina et al. [10,16,19].

RETRACTED

The demographic analysis in our study revealed several concerning trends. The higher resistance rates observed in younger patients (aged 21-30 years) may reflect greater antibiotic exposure in this age group. The urban-rural disparity in resistance patterns, with urban residents showing significantly higher resistance rates, suggests potential differences in antibiotic access and usage patterns between these populations. These findings emphasize the need for targeted interventions in urban areas where antibiotic use may be less regulated.

The relationship between prior antibiotic exposure and resistance patterns merits particular attention. The progressive increase in resistance rates with multiple antibiotic exposures underscores the importance of judicial antibiotic use and effective antibiotic stewardship programs. Similarly, the correlation between illness severity, duration of hospital stay, and resistance rates highlights the complex interplay between healthcare exposure and the development of antibiotic resistance.

Our findings regarding hospital stay duration and resistance patterns raise important questions about healthcare-associated resistance development. The progressive increase in resistance rates with longer hospital stays suggests potential nosocomial factors in resistance development, though the current study design cannot establish causality in this relationship.

The study's findings have immediate clinical implications for the treatment of typhoid fever in endemic regions. The superior effectiveness of meropenem suggests its preferential use when carbapenem therapy is indicated. However, the overall high resistance rates across all tested carbapenems emphasize the need for careful antibiotic selection based on local resistance patterns and individual patient factors.

Strengths and limitations

This research derives its strength from several key methodological aspects. The large sample size of 626 isolates, collected over a two-year period, provides robust statistical power and temporal representation of resistance patterns. The standardized testing methodology, employing validated protocols and quality control measures, ensures the reliability of the findings. The comprehensive demographic and clinical data collection allows for detailed analysis of resistance patterns across various patient subgroups, contributing to the study's clinical relevance.

RETRACTED

However, several limitations warrant consideration when interpreting these results. The single-center nature of the study may limit the generalizability of findings to other geographic regions or healthcare settings. The absence of molecular resistance mechanism analysis prevents deeper understanding of the genetic basis for observed resistance patterns. The study's exclusion of the pediatric population restricts its applicability across all age groups, while the limited clinical outcome data constrains our ability to correlate resistance patterns with treatment outcomes. Additionally, the potential for selection bias in a hospital-based study should be considered when extrapolating these findings to community settings. The cross-sectional design, while appropriate for prevalence estimation, cannot establish causal relationships between observed factors and resistance development.

## Conclusions

This study demonstrates a concerning pattern of carbapenem resistance in *S.* Typhi isolates, with meropenem showing the highest efficacy (42.7% sensitivity) among the tested carbapenems, followed by ertapenem (35.5%) and doripenem (11.98%). The high resistance rates observed, particularly for doripenem, highlight the urgent need for alternative treatment strategies and ongoing monitoring of resistance patterns. The progressive relationship between healthcare exposure and resistance development emphasizes the importance of antimicrobial stewardship programs and the need for evidence-based prescribing practices. Based on our findings, we recommend several specific clinical practice modifications for regions with high MDR *S.* Typhi prevalence. These include implementation of mandatory antibiotic sensitivity testing before initiating carbapenem therapy, consideration of meropenem as the preferred carbapenem when indicated, development of institutional protocols for combination therapy approaches, regular monitoring and reporting of resistance patterns, and institution of formal antibiotic stewardship programs. The observed resistance patterns suggest the urgent need for novel therapeutic approaches, including the investigation of new antibiotic combinations, the development of alternative treatment strategies, and the implementation of preventive measures to limit further resistance development.

These findings suggest that clinicians in regions with high resistance rates should carefully consider their choice of carbapenem, with meropenem potentially offering the best therapeutic option when indicated. However, the overall high resistance rates across all tested carbapenems underscore the critical need for new therapeutic approaches and more effective infection prevention strategies.
